This article has been retracted.

# Diagnostic Performance of Atherosclerotic Carotid Plaque Neovascularization with Contrast-Enhanced Ultrasound: A Meta-Analysis

**DOI:** 10.1155/2022/7531624

**Published:** 2022-03-07

**Authors:** Shanshan Dong, Jianzhong Hou, Caiyun Zhang, Guilin Lu, Wenjuan Qin, Lei Huang, Guangqin Zhou

**Affiliations:** ^1^Department of Function, First Affiliated Hospital, School of Medical, Shihezi University, Shihezi, Xinjiang 832000, China; ^2^Department of General Surgery, First Affiliated Hospital, School of Medical, Shihezi University, Shihezi, Xinjiang 832000, China

## Abstract

**Objectives:**

To evaluate the diagnostic performance of contrast-enhanced ultrasound (CEUS) for atherosclerotic carotid plaque neovascularization.

**Methods:**

The electronic databases like PubMed, Embase, OVID, and Web of Science were used to search for the relevant studies, which are involved in the evaluation of the diagnostic parameters of QUS for atherosclerotic carotid plaque neovascularization. Review Manager 5.4 and Stata 14.0 were used to estimate the pooled diagnostic value of CEUS. Forest plots, sensitivity analysis, and Deeks' funnel plots were performed on the included studies.

**Results:**

Ten studies eventually met the final inclusion criteria. For diagnostic performance, CUES showed that the pooled values of sensitivity, specificity, positive likelihood odds ratios, negative likelihood odds ratios, and diagnostic odds ratios were 0.83 (95% CI 0.78-0.86), 0.77 (95% CI 0.68-0.84), 3.61 (95% CI 2.59-5.03), 0.23 (95% CI 0.18-0.28), and 16.02 (95% CI 10.02-25.60), respectively. The estimate of the area under curve (AUC) was 0.85 (95% CI 0.82-0.88).

**Conclusion:**

Our research supported that CEUS had high sensitivity and specificity in the diagnosis of atherosclerotic carotid plaque neovascularization. More high-quality prospective multicenter studies focusing on the accuracy of CEUS for carotid atherosclerotic plaque should be performed to verify our conclusions.

## 1. Introduction

Atherosclerotic disease is a systemic disease of the arterial wall, which may be a form of cardiovascular inflammatory disease [1]. There are many theories about its pathogenesis, but at present, the main theory is that the arterial wall is a chronic response to endothelial cell injury, which promotes the progress of the disease through the interaction of oxidized lipoproteins, macrophages, T cells, and normal cell components of the arterial wall [2–4].

With the development of atherosclerosis, various local and systemic factors will promote neovascularization. Neovascularization in plaque (IPN) is one of the important characteristics of vulnerable plaque formation [5, 6]. Due to the lack of support of vascular smooth muscle cells and endothelial cells, vascular fragility, high permeability, white blood cells, and red blood cells exudate, leading to bleeding in plaque [7, 8]. Fleiner et al.'s study have confirmed that the presence and degree of neovascularization in vulnerable plaques are related to plaque rupture and clinical cardiovascular and cerebrovascular events, which can increase the risk of sudden cardiovascular and cerebrovascular events, such as stroke, transient ischemic attack, and myocardial infarction [9].

Therefore, early assessment of the stability of carotid atherosclerotic plaque and prediction of the risk of plaque rupture have great significance for the prevention of cardiovascular and cerebrovascular events and the development of treatment programs [8, 10]. In clinical practice, the carotid artery is usually selected as the detection path to evaluate the characteristics of atherosclerotic plaque [11, 12]. B-ultrasound and color Doppler are commonly used in the diagnosis of carotid atherosclerotic plaque formation and stenosis [13, 14]. Feinstein first reported the feasibility of using contrast-enhanced ultrasound (CEUS) to identify IPN. Recently, a number of studies have shown that CEUS can significantly improve the imaging effect of IPN [15].

Perfluoroxide microbubbles (a kind of good vascular tracer) are used for CEUS, which was injected through the elbow vein, supplemented by normal saline, targeted and nontargeted development [4]. The neovascularization in plaque was analyzed qualitatively and quantitatively by a 4~10 MHz linear array probe and contrast software harmonic imaging.

Although many studies have reported the application results of CEUS in the evaluation of neovascularization in carotid plaques, in view of the variability of the reported results, we conducted a meta-analysis of relevant studies, so as to obtain the preliminary evidence for the feasibility of CEUS in the diagnosis of neovascularization in carotid plaques.

## 2. Methods

### 2.1. Literature Search Strategy

A systematic search for eligible studies from January 2000 to May 2021 was conducted on PubMed, Embase, OVID, and Web of Science with relevant keywords: (1) atherosclerotic carotid plaque, (2) neovascularization, and (3) contrast-enhanced ultrasound are the keywords used in combination with the Boolean operators “AND” or “OR” to search literature. There were no restrictions on the language of publication in the literature search. In order to maximize the specificity and sensitivity of the retrieval, the author should also refer to the list of references retrieved to look for other retrieval strategies that have not been found in related studies.

### 2.2. Study Selection

We included articles that met the following inclusion criteria:

1. Patients with arterial stenosis and/or ischemic attack
2. Study outcomes with available data as follow: true positive (TP), false positive (FP), false negative (FN), and true negative (TN)
3. Patients in which the diagnosis of neovascularization in carotid atherosclerotic plaques was based on the gold standard, such as pathological or clinical diagnosis
4. Full text was available

We excluded the study for the following reasons:

1. Studies that did not meet the inclusion criteria
2. Relevant results were not reported or cannot be used
3. Review, abstract, or duplicate publication

### 2.3. Data Extraction

A panel of two reviewers independently screened all titles and abstracts identified by a literature search, obtained full-text articles from all potentially eligible studies, assessed their eligibility, and extracted the following data from each eligible study: first author's name, year of publication, country of origin, language, sample size, disease, patient's age and gender, test location, reference standard, and primary outcome (TP, FP, FN, and TN).

### 2.4. Quality Assessment

Two reviewers assessed the quality of individual trials using the diagnostic accuracy study quality assessment (QUADAS) criteria recommended by the Cochrane Diagnostic Test Accuracy Working Group. There were 14 standards in QUADAS, which was evaluated one by one with “yes,” “no,” or “unclear”. Any differences in domain assignments were resolved by consensus.

### 2.5. Statistical Analysis

Meta-analysis was performed with Review Manager 5.4 and Stata 14.0. The chi square test and *I*^2^ statistics were used to test the heterogeneity. If *I*^2^ < 50% and *P* < 0.05, the homogeneity of the included literature was considered to be good and the fixed-effects model was used; if *I*^2^ > 50% or *P* ≥ 0.05, it was considered that there was heterogeneity between the studies, the random-effects model was used, and sensitivity analysis was conducted to evaluate the robustness of the results. Deeks' funnel plot would be used to identify publication bias, and *P* > 0.05 was considered indicative of no significant publication bias.

## 3. Results

### 3.1. Search Process

A total of 752 studies were identified by electronic search. After careful reading, 110 studies meeting the inclusion criteria were identified. Among them, 100 were further excluded due to different research designs or insufficient data. Finally, 10 papers were included in this meta-analysis [16–25]. Further information about the search process and inclusion and exclusion criteria was shown in Figure 1.

### 3.2. Characteristics of Included Studies

The characteristics of 10 studies that were included in our meta-analysis were presented in Table 1. The published years were between 2007 and 2020. These studies contained a total of 825 patients with arterial stenosis and/or ischemic attack. Among the studies, all studies were published in the English language, seven studies were from China, and the other three were from the USA, the UK, and Italy. Seven studies used pathology as the reference standard, while 3 adopted clinic diagnosis as the gold standard.

### 3.3. Results of Quality Assessment

According to the QUADAS-2 tool, the methodological quality of included studies was evaluated for the bias risk and clinical applicability. As shown in Figure 2, three studies showed high risk of the reference standard, because they chose clinical symptoms for the reference standard, which existed a certain uncertainty. One article showed high risk of patient selection. The summary of bias risk and applicability concerns of the 10 included studies was illustrated in Figure 3.

### 3.4. Results of Diagnostic Accuracy

Meta-analysis was conducted, and the overall pooled sensitivity and specificity were 0.83 (95% CI [0.78, 0.86], *I*^2^ = 2.04%, *P* = 0.42, fixed-effects model) and 0.77 (95% CI [0.68, 0.84], *I*^2^ = 71.11%, *P* < 0.001, random-effects model), respectively (Figure 4). The pooled PLR, NLR, and DOR were 3.61 (95% CI [2.59, 5.03], *I*^2^ = 47.77%, *P* < 0.001, random-effects model), 0.23 (95% CI [0.18, 0.28], *I*^2^ = 0%, *P* = 0.55, fixed-effects model), and 16.02 (95% CI [10.02, 25.60], *I*^2^ = 90.44%, *P* < 0.001, random-effects model), respectively (Figures 5, 6). The area under the curve was 0.85 (95% CI [0.82, 0.88]) (Figure 7).

### 3.5. Results of Heterogeneity Analysis

The Spearman correlation coefficient was 0.304 (*P* = 0.393), suggesting that no obvious heterogeneity and threshold effect was found. No significant heterogeneity was found in sensitivity (*I*^2^ = 2.04%, *P* = 0.42) and NLR (*I*^2^ = 0%, *P* = 0.55). However, heterogeneity was detected in specificity (*I*^2^ = 71.11%, *P* < 0.001), PLR (*I*^2^ = 47.77%, *P* < 0.001), and DOR (*I*^2^ = 90.44%, *P* < 0.001); therefore, the random-effects model was performed.

### 3.6. Sensitivity Analysis

Sensitivity analysis was performed to assess the stability of the results by removing one study at a time and iteratively recalculating the key outcome measures, and there were no articles that unduly influenced the findings, and they did not change obviously, indicating that the heterogeneity of these studies was relatively stable.

### 3.7. Publication Bias

To assess for any evidence of publication bias among the included studies, Deeks' funnel plots were performed. The *P* value was 0.83, which indicated that no obvious publication bias existed in this meta-analysis. (Figure 8).

## 4. Discussion

Some studies had showed that ultrasound has higher sensitivity and accuracy in detecting plaque instability than color Doppler [26–28], such as in Ten et al.'s study, the sensitivity of ultrasound in plaque detection was 88% and specificity was 72%, while the sensitivity of color Doppler was 29% and specificity was 54% [29]. Ultrasound can better distinguish the internal and middle membrane boundaries of the carotid artery and find and identify the integrity of the fibrous cap on the plaque surface, which played an important role in clinical application [30–32].

Ritter et al. performed ipsilateral intracranial microemboli signal detection in 41 patients with symptomatic carotid atherosclerosis and performed contrast-enhanced ultrasound 30 minutes later to evaluate the neovascularization in plaque [33]. It was found that the intracranial microemboli were linearly correlated with neovascularization in symptomatic carotid atherosclerotic plaque. Deyama et al. found that the more complex and larger coronary artery lesions and higher prevalence of multivessel coronary heart disease and chronic total occlusion coronary artery lesions would lead to a higher score of CEUS in evaluating neovascularization in carotid plaque [34]. At the same time, they also found that after taking statins, the visual score of contrast-enhanced ultrasound intensity of patients will decrease. They believe that statins can reduce the neovascularization in plaque and inhibit the development of adventitial nutrient vessels and atherosclerosis. Therefore, CEUS can be used to evaluate the clinical efficacy of drugs and monitor the progress of nutrient vessels and plaque [35–37].

Our meta-analysis mainly found that the sensitivity of CEUS in the diagnosis of carotid atherosclerotic plaque neovascularization was 68% and specificity was 78%, indicating that the underdiagnosis rate was 32% and the misdiagnosis rate was 22%. The DOR was 9.47, which indicated that CEUS had a high accuracy in identifying neovascularization in atherosclerotic plaque. The results of this study also showed that the sensitivity of CEUS has a small range (0.63~0.73) in the diagnosis population, suggesting that the diagnosis was stable. The AUC was 0.8346, which indicated that the diagnostic efficiency was relatively high. Tang et al.'s study found that the detection rate of neovascularization in carotid atherosclerotic plaque by ultra-microangiography was slightly higher than that by CEUS but the difference was not statistically significant [32].

The heterogeneity among the 10 studies may be related to the following factors: (1) the degree of carotid artery stenosis selected in each study was different, (2) these studies used different contrast agents, and (3) they used different mechanical index values. These factors suggested that CEUS needs to improve the standardization of test methods to ensure reliability and repeatability and it can be effectively integrated into clinical practice in this way.

There were some limitations in this study. First of all, because the operator's experience and skills had a certain impact on the results of ultrasound diagnosis, subjective factors and operator's experience had a great influence on the visual score of neovascularization in plaque [38, 39]. Secondly, in the included studies, pathology or clinical symptoms were selected as the gold standard and inconsistent standards may affect the judgment of sensitivity and specificity.

In conclusion, CEUS had high sensitivity and specificity in the diagnosis of IPN with obvious advantages. We believe that with the development of science and technology and in-depth research, CEUS will plays a greater role in the evaluation of atherosclerotic plaque. In view of the limitations of CEUS, the accuracy of CEUS in the diagnosis of carotid atherosclerotic plaque needed to be further verified by more high-quality prospective multicenter studies.

## Figures and Tables

**Figure 1:** Flow diagram of the evidence search and selection process.

**Figure 2:** The quality assessment for included studies: low risk (green), unclear (yellow), and high risk (red).

**Figure 3:** Summary of bias assessments for each included studies.

**Figure 4:** Forest plot: sensitivity and specificity of CEUS.

**Figure 5:** Forest plot: PLR and NLR of CEUS.

**Figure 6:** Forest plot: DOR of CEUS.

**Figure 7:** Forest plot: SROC and AUC of CEUS.

**Figure 8:** Deeks' funnel plot for evaluating potential publication bias.

**Table 1:** Characteristics of the included studies.

Study	Country	Language	Disease	No. participants	Gender (M/F)	Age	Reference standard	TP	FP	FN	TN
[22]	USA	English	Arterial stenosis (≥50%)	17	10/7	/	Pathology	5	2	2	8
[24]	China	English	Ischemic attack and/or cerebrovascular ischemic stroke	104	83/21	62 ± 9	Pathology	36	14	13	41
[16]	China	English	Ischemic stroke	176	100/76	62 ± 7	Clinic diagnosis	56	22	12	86
[19]	UK	English	Arterial stenosis (>30%)	37	27/10	69.9 ± 8.5	Clinic diagnosis	12	3	4	18
[25]	China	English	Arterial stenosis (≥50%)	46	43/3	62 ± 7	Clinic diagnosis	15	15	2	14
[17]	Italy	English	Arterial stenosis (≥70%)	50	28/22	69.9 ± 7.3	Pathology	32	5	2	11
[23]	China	English	Carotid atherosclerotic plaques	93	78/15	62.5 (50, 91)	Pathology	28	22	5	38
[21]	China	English	Acute coronary syndrome and stable coronary artery disease	120	39/21	62.8 ± 9.2	Pathology	36	9	9	66
[18]	China	English	Arterial stenosis (≥60%)	131	/	/	Pathology	56	7	12	24
[20]	China	English	Ischemic stroke	51	43/8	67.0 ± 6.5	Pathology	21	2	2	26

TP: true positive; FP: false positive; FN: false negative; TN: true negative.

## Data Availability

No data were used to support this study.

## References

[1] Kim H. S., Woo J. S., Kim B. Y. (2014). Biochemical and clinical correlation of intraplaque neovascularization using contrast-enhanced ultrasound of the carotid artery. *Atherosclerosis*.

[2] Caplice N. M., Martin K. (2010). Contrast-enhanced ultrasound and the enigma of plaque neovascularization^*^. *JACC: Cardiovascular Imaging*.

[3] Deng Y. B., Zhu Y., Liu Y. N., Bi X. J., Bi X. J. (2009). 0015: Contrast-enhanced ultrasound imaging of carotid plaque neovascularization: correlation with clinical symptoms. *Ultrasound in Medicine & Biology*.

[4] van den Oord S. C. H., Akkus Z., Bosch J. G. (2015). Quantitative contrast-enhanced ultrasound of intraplaque neovascularization in patients with carotid atherosclerosis. *Ultraschall in der Medizin*.

[5] Van Den Oord S. C., Akkus Z., Renaud G. (2014). Assessment of carotid atherosclerosis, intraplaque neovascularization, and plaque ulceration using quantitative contrast-enhanced ultrasound in asymptomatic patients with diabetes mellitus. *European Heart Journal Cardiovascular Imaging*.

[6] Hagiwara Y., Ogura H., Shimizu T., Imai H., Hasegawa J., Hasegawa Y. (2018). Transoral carotid ultrasonography with superb microvascular imaging. *Neurosonology*.

[7] Evdokimenko A., Druina L., Druina L. (2017). Characteristics of carotid plaques neovascularization and the resolution power of contrast-enhanced ultrasound to detect intraplaque microvessels. *Cerebrovascular Diseases*.

[8] Schmidt C., Fischer T., Rückert R. I. (2017). Identification of neovascularization by contrast–enhanced ultrasound to detect unstable carotid stenosis. *PLoS One*.

[9] Fleiner M., Kummer M., Mirlacher M. (2004). Arterial neovascularization and inflammation in vulnerable patients: early and late signs of symptomatic atherosclerosis. *Circulation*.

[10] Decano J. L., Moran A. M., Ruiz-Opazo N., Herrera V. L. M. (2011). Molecular imaging of vasa vasorum neovascularization via DEspR-targeted contrast-enhanced ultrasound micro-imaging in transgenic atherosclerosis rat model. *Molecular Imaging & Biology*.

[11] Cattaneo M., Staub D., Porretta A. P. (2016). Contrast-enhanced ultrasound imaging of intraplaque neovascularization and its correlation to plaque echogenicity in human carotid arteries atherosclerosis. *International Journal of Cardiology*.

[12] Nakamura J., Nakamura T., Deyama J. (2015). Assessment of carotid plaque neovascularization using quantitative analysis of contrast-enhanced ultrasound imaging is useful for risk stratification in patients with coronary artery disease. *International Journal of Cardiology*.

[13] Van D. (2012). Semi-automated quantification of intraplaque neovascularization using contrast-enhanced ultrasound of the carotid arteries.

[14] Zhang Q., Li C., Zhou M. (2015). Quantification of carotid plaque elasticity and intraplaque neovascularization using contrast-enhanced ultrasound and image registration-based elastography. *Ultrasonics*.

[15] Feinstein S. B. (2006). Contrast ultrasound imaging of the carotid artery vasa vasorum and atherosclerotic plaque neovascularization. *Journal of the American College of Cardiology*.

[16] Huang P. T., Chen C. C., Aronow W. S. (2010). Assessment of neovascularization within carotid plaques in patients with ischemic stroke. *World Journal of Cardiology*.

[17] Iezzi R., Petrone G., Ferrante A. (2015). The role of contrast-enhanced ultrasound (CEUS) in visualizing atherosclerotic carotid plaque vulnerability: which injection protocol? Which scanning technique?. *European Journal of Radiology*.

[18] Ning B., Zhang D., He W., Wang L. S., Jin Z. Q. (2019). A study on distribution features of neovascularization in atherosclerotic carotid artery plaques: comparing contrast-enhanced ultrasound with histopathology. *Ultrasonic Imaging*.

[19] Owen D. R., Shalhoub J., Miller S. (2010). Inflammation within carotid atherosclerotic plaque: assessment with late-phase contrast-enhanced US. *Radiology*.

[20] Lyu Q., Tian X., Ding Y. (2021). Evaluation of carotid plaque rupture and neovascularization by contrast-enhanced ultrasound imaging: an exploratory study based on histopathology. *Translational Stroke Research*.

[21] Qin C., Zhang L., Wang X., Duan Y., Ye Z., Xie M. (2018). Evaluation of carotid plaque neovascularization in patients with coronary heart disease on contrast-enhanced ultrasonography. *Journal of Ultrasound in Medicine*.

[22] Shah F., Balan P., Weinberg M. (2007). Contrast-enhanced ultrasound imaging of atherosclerotic carotid plaque neovascularization: a new surrogate marker of atherosclerosis?. *Vascular Medicine*.

[23] Sun X., Wang J., Wu X. L., Xu H. Y., Xing Y. Q., Yang F. (2016). Evaluation of the stability of carotid atherosclerotic plaque with contrast-enhanced ultrasound. *Journal of Medical Ultrasonics*.

[24] Xiong L., Deng Y. B., Zhu Y., Liu Y. N., Bi X. J. (2009). Correlation of carotid plaque neovascularization detected by using contrast-enhanced US with clinical symptoms. *Radiology*.

[25] Zhou Y., Xing Y., Li Y. (2013). An assessment of the vulnerability of carotid plaques: a comparative study between intraplaque neovascularization and plaque echogenicity. *BMC Medical Imaging*.

[26] Staub D., Partovi S., Schinkel A. F. (2011). Correlation of carotid artery atherosclerotic lesion echogenicity and severity at standard US with intraplaque neovascularization detected at contrast-enhanced US. *International Journal of Medical Radiology*.

[27] Partovi Sasan, Loebe Matthias, Aschwanden Markus (2012). Contrast-enhanced ultrasound for assessing carotid atherosclerotic plaque lesions. *American Journal of Roentgenology*.

[28] Filis K., Toufektzian L., Galyfos G. (2017). Assessment of the vulnerable carotid atherosclerotic plaque using contrast-enhanced ultrasonography. *Vascular*.

[29] Ten Kate G. L., van Dijk A. C., van den Oord S. C. H. (2013). Usefulness of contrast-enhanced ultrasound for detection of carotid plaque ulceration in patients with symptomatic carotid atherosclerosis. *American Journal of Cardiology*.

[30] Schinkel A., Bosch J. G., Staub D., Adam D., Feinstein S. B. (2020). Contrast-enhanced ultrasound to assess carotid intraplaque neovascularization. *Ultrasound in Medicine & Biology*.

[31] Shah B. N., Gujral D. M., Chahal N. S., Harrington K. J., Nutting C. M., Senior R. (2016). Plaque neovascularization is increased in human carotid atherosclerosis related to prior neck radiotherapy: a contrast-enhanced ultrasound study. *Jacc Cardiovascular Imaging*.

[32] Tang J., Ultrasound D. O., Hospital X. C. (2019). Application value of superb microvascular imaging and contrast-enhanced ultrasound in neovascularization of carotid plaques with different thickness. *Chinese Journal of CT and MRI*.

[33] Ritter M. A., Theismann K., Schmiedel M., Ringelstein E. B., Dittrich R. (2013). Vascularization of carotid plaque in recently symptomatic patients is associated with the occurrence of transcranial microembolic signals. *European Journal of Neurology*.

[34] Deyama J., Nakamura T., Takishima I. (2013). Contrast-enhanced ultrasound imaging of carotid plaque neovascularization is useful for identifying high-risk patients with coronary artery disease. *Circulation Journal*.

[35] Yan H., Wu X., He Y., Staub D., Wen X., Luo Y. (2021). Carotid Intraplaque neovascularization on contrast-enhanced ultrasound correlates with cardiovascular events and poor prognosis: a systematic review and meta-analysis. *Ultrasound in Medicine & Biology*.

[36] Hoogi A., Adam D., Hoffman A., Kerner H., Reisner S., Gaitini D. (2011). Carotid plaque vulnerability: quantification of neovascularization on contrast-enhanced ultrasound with histopathologic correlation. *AJR. American Journal of Roentgenology*.

[37] Hou X. X., Chu G. H., Yu Y. (2018). Prospects of contrast-enhanced ultrasonography for the diagnosis of peripheral arterial disease: a meta-analysis. *Journal of Ultrasound in Medicine*.

[38] Kunte H., Schmidt C., Harms L., Ruckert R. I., Grigoryev M., Fischer T. (2012). Contrast-enhanced ultrasound and detection of carotid plaque neovascularization. *Neurology*.

[39] Li C., He W., Guo D. (2014). Quantification of carotid plaque neovascularization using contrast-enhanced ultrasound with histopathologic validation. *Ultrasound in Medicine & Biology*.

